The article "The miR-491-3p/mTORC2/FOXO1 regulatory loop modulates chemo-sensitivity in human tongue cancer" was published in 2015. Journal: Oncotarget.

# The miR-491-3p/mTORC2/FOXO1 regulatory loop modulates chemo-sensitivity in human tongue cancer

**DOI:** 10.18632/oncotarget.3165

**Published:** 2015-02-19

**Authors:** Guopei Zheng, Xiaoting Jia, Cong Peng, Yingen Deng, Jiang Yin, Zhijie Zhang, Nan Li, Min Deng, Xiaorong Liu, Hao Liu, Minying Lu, Chengkun Wang, Yixue Gu, Zhimin He

**Affiliations:** ^1^ Cancer Hospital and Cancer Research Institute of Guangzhou Medical University, Guangzhou 510095, Guangdong, China

**Keywords:** tongue cancer, miR-491-3p, Rictor, mTORC2, drug resistance

## Abstract

We found that levels of miR-491-3p were decreased in multidrug-resistant tongue cancer (TC) cells. Induction of miR-491-3p expression sensitized TC cells to chemotherapy. In agreement, functional inhibition of miR-491-3p enhanced resistance of TC cells to chemotherapy. We found that miR-491-3p directly targeted mTORC2 component Rictor and inhibited mTORC2 activity, which was increased in resistant TC cells with high p-Akt(Ser473), p-SGK1(Ser422) and p-FOXO1(Thr24) levels. Inhibition of mTORC2 activity via either Rictor knockdown or mTOR inhibitor in turn sensitized TC cells to chemotherapy. In agreement, overexpression of Rictor increased the mTORC2 activity and induced resistance of TC cells to chemotherapy. As a feedback loop, mTORC2 downregulated miR-491-3p expression by inactivating FOXO1, which otherwise would transcriptionally induce miR-491-3p expression. Levels of miR-491–3 and Rictor or mTORC2 activity negatively correlated in TC tissues. Finally, low levels of miR-491-3p and highly expressed Rictor were associated with poor prognosis in tongue cancer patients. These data provide a rationale for targeted intervention on miR-491-3p/mTORC2 axis to enhance the efficacy of chemotherapy against tongue cancer.

## INTRODUCTION

Tongue cancer is the most common oral cancer. In United States alone, it has been estimated 12,060 new cases and 2030 deaths from tongue cancer in 2011 [1]. Tongue cancer frequently metastasizes and has a poorer prognosis than carcinoma of other sites in the oral cavity. In the clinic, tongue cancer usually leads to malfunction of mastication, speech and deglutition. Chemotherapy alone or its combination with local/regional treatment is effective for reducing tumor size, inhibiting distant metastasis, preserving organ function and prolonging patient survival [2]. However, the efficacy of chemotherapy is usually attenuated due to intrinsic and/or acquired drug resistance. A large proportion of chemo-resistant tongue cancers show more aggressive tumor behavior and an even worse clinical outcome [3, 4]. While multiple mechanisms, such as insensitivity to drug-induced apoptosis, increased DNA repair and induction of drug-detoxifying mechanisms, have been proposed to play an important role in the development of cancer drug resistance [5], the precise causes of chemotherapy resistance in tong cancer remain elusive.

The article "The miR-491-3p/mTORC2/FOXO1 regulatory loop modulates chemo-sensitivity in human tongue cancer" was published in 2015. Journal: Oncotarget.

Recently, both basic research and clinical studies demonstrate a critical role for miRNAs in chemotherapy resistance [6]. miRNAs typically function in the post-transcriptional regulation of genes by binding to the 3′-untranslated region (3′UTR) of target messenger RNA (mRNA), which leads to translational repression or mRNA degradation [7]. It has been shown that miRNAs regulate a wide variety of physiological and pathological processes, including development, differentiation, proliferation, stress response, metabolism and apoptosis. miRNAs could function as both tumor suppressors and tumor promoters in cancer [8]. With regard to cancer treatment, some studies have suggested that selected miRNAs may influence the response of cancer cells to chemotherapy [9]. Specific miRNAs have been shown an altered expression in drug-resistant cancer cells. For example, miR-34a was downregulated in drug-resistant prostate cancer cells, and ectopic expression of miR-34a resulted in growth inhibition and sensitized the cells to camptothecin [10]; in addition, miR-200b expression was significantly downregulated in docetaxel-resistant NSCLC cells [11]. Furthermore, miRNAs also modulate the process of EMT (epithelial-mesenchymal transition) and cancer stem cell program. For example, Adam et al. showed that miR-200 regulated the EMT in bladder cancer cells and reversed the resistance to EGFR inhibitor therapy [12]. A study by Li et al. revealed that the re-expression of the miR-200 family inhibited EMT and increased the sensitivity of pancreatic cancer cells to gemcitabine [13]. Thus, studies to further understand the role of miRNAs in cancer drug resistance may facilitate the development of innovative strategies for cancer treatment.

There are limited reports regarding the role of miRNA in tongue carcinogenesis and drug response. Wong et al. showed that miR-184 was overexpressed in tongue squamous cell carcinoma (TSCC), and the reduction of miR-184 inhibited cell proliferation and induced apoptosis through c-Myc downregulation [14]. Li et al. reported that miR-21 was overexpressed in TSCC relative to the adjacent normal tissues, and miR-21 inhibition induced cell growth inhibition and apoptosis *in vitro* and *in vivo* [15]. Recently, Sun et al. found that re-overexpression of miR-200b and miR-15b in cisplatin-resistant tongue cancer cells reduced BMI1 expression, and thereby sensitized the cells to chemotherapy [16]. In the present study, we screened for miRNAs with differential expression in acquired multidrug-resistant TSCC cells (Tca8113/PYM) [17] as compared to the sensitive parent cell line Tca8113. We found that miR-491-3p was significantly downregulated in Tca8113/PYM cells. Importantly, restored expression of miR-491-3p re-sensitized Tca8113/PYM cells to the treatment of PYM and cisplatin (cDDP). Conversely, inhibition of miR-491-3p reduced the sensitivity of Tca8113, SCC-25 and CAL-27 cells to chemotherapy. MiR-491-3p appeared to exert its effect via regulating Rictor expression in mTORC2 complex. Furthermore, we demonstrated the expression of miR-491-3p could be transcriptionally regulated by FOXO1, which was inactivated by mTORC2. Our data suggest a negative regulatory loop between mTORC2 signaling and miR-491-3p mediated by FOXO1 in chemo-resistant tong cancer cells.

The article "The miR-491-3p/mTORC2/FOXO1 regulatory loop modulates chemo-sensitivity in human tongue cancer" was published in 2015. Journal: Oncotarget.

## RESULTS

### Identification of differentially expressed miRNAs between Tca8113/PYM and Tca8113 cells

To investigate whether miRNAs are involved in the PYM-induced multidrug resistance in tong cancer, the miRNA expression profiles in Tca8113/PYM cells and its parent cell line Tca8113 were compared by miRNA microarray analysis. Thirty seven (37) differentially expressed miRNAs were identified using a cutoff value of 2-fold change between the two cell lines. Of these 37 miRNAs, 25 were upregulated and 12 were downregulated in Tca8113/PYM cells (Figure 1A). The data were further confirmed by qRT-PCR analysis. Nine miRNAs were examined, and a good correlation between the qRT-PCR results and the microarray data was observed (Figure 1B).

**Figure 1:** Differential expression of miRNAs between Tca8113 and Tca8113/PYM cells **(A)** miRNA microarray showed the differential expression of miRNAs, with the fold change as the ratio of Tca8113/PYM to Tca8113. **(B)** Validation of the microarray results using miRNA-specific qRT-PCR. The relative expression of the selected miRNAs is shown as the fold difference between Tca8113/PYM and Tca8113 cells by normalizing to RNU6 as endogenous control. **(C)** miR-491-3p expression pattern in tongue cancer cell lines detected by qRT-PCR and the expression level in Tca8113 was set as 1, *vs* Tca8113, *p < 0.01. Columns: the relative ratio of miRNA expression to Tca8113; Bars: SD from three independent assays.

### miR-491-3p modulates chemosensitivity in tongue cancer cells

MiR-491-3p expression was significantly down regulated in the chemo-resistant Tca8113/PYM cells. To investigate whether the reduction of miR-491-3p played a causal role in the development of drug resistance, we used a gain- or loss-of-function approach in a series of tongue cancer cell lines. As shown in Figure 1C, miR-491-3p expression was relatively higher in chemo-sensitive SCC-25 and CAL-27 tongue cancer cell lines than that in Tca8113/PYM cells. Increased miR-491-3p via transfection of miR-491-3p mimics significantly enhanced the sensitivity of Tca8113/PYM cells to PYM- and cDDP-induced growth inhibition and apoptosis (Figure 2A). Inversely, the sensitivity of Tca8113 (Figure 2B), SCC-25 (Figure 2C) and CAL-27 (Figure 2D) cells to PYM or cDDP was dramatically decreased upon inhibition of miR-491-3p with specific inhibitor, accompanied with reduced apoptosis-induced by PYM or cDDP.

The article "The miR-491-3p/mTORC2/FOXO1 regulatory loop modulates chemo-sensitivity in human tongue cancer" was published in 2015. Journal: Oncotarget.

**Figure 2:** miR-491-3p sensitized tongue cancer cells to chemotherapy **(A)** overexpressed miR-491-3p via transfection of miR-491-3p mimics sensitized Tca8113/PYM cells to PYM and cDDP, detected by MTS assay to determing proliferation and hochest stain to determining apoptosis respectively. **(B–D)** functional inhibition of miR-491-3p with specific inhibitor attenuated the sensitivity of Tca8113, SCC-25 and CAL-27 cell lines to PYM and cDDP, detected by MTS assay and hochest stain respectively.

### miR-491-3p directly targets Rictor, a component of mTORC2 complex

We next used miRNA database TargetScan (http://www.targetscan.org) to predict potential targets of miR-491-3p. The mTORC2 component Rictor with a conserved binding site of miR-491-3p was selected for further identification (Figure 3A). There was no significant difference of the *Rictor* mRNA level in selected cell lines (Figure 3B). However, the Rictor protein level in Tca8113/PYM cells was much higher than that in Tca8113, SCC-25 and CAL-27 cell lines (Figure 3C). Notably, transfection with miR-491-3p mimics significantly downregulated Rictor protein level in Tca8113/PYM cells, and the miR-491-3p inhibitor clearly upregulated Rictor protein level in Tca8113, SCC-25 and CAL-27 cell lines (Figure 3D). To assess whether Rictor is a direct target of miR-491-3p, a luciferase reporter vector containing the putative Rictor 3′UTR target site for miR-491-3p (pMir-Wt, as wildtype version) or a mutant version with a deletion of 7bp in the seed sequence was constructed (pMir-Mut). As shown, in Tca8113, SCC-25 and CAL-27 cell lines, the luciferase activities from mutant version were higher than that from wildtype version. In contrast the luciferase activity from wildtype version in Tca8113/PYM cells was higher than that in Tca8113, SCC-25 and CAL-27 cells (Figure 3E), suggesting that endogenous miR-491-3p inhibits Rictor expression by binding to the seed sequence in the 3′UTR of *Rictor* mRNA. Moreover, miR-491-3p mimics significantly repressed the luciferase activity of the vector with wild-type Rictor 3′UTR in Tca8113/PYM cells, but the mutant version abrogated the repressive ability of miR-491-3p (Figure 3F). Inversely, miR-491-3p inhibitor increased the luciferase activities from the wildtype version, and the mutant version abrogated the facilitative effect of miR-491-3p inhibitor (Figure 3F). These results strongly demonstrated the specificity of miR-491-3p targeting *Rictor* mRNA.

The article "The miR-491-3p/mTORC2/FOXO1 regulatory loop modulates chemo-sensitivity in human tongue cancer" was published in 2015. Journal: Oncotarget.

**Figure 3:** miR-491-3p repressed Rictor protein expression **(A)** Schematic of predicted miR-491-3p site in the 3′UTR of human Rictor mRNA, which broadly conserved among vertebrates. **(B)** The expression pattern of Rictor in mRNA levels in selected cell lines detected by qRT-PCR by normalizing to GAPDH as endogenous control and the expression level in Tca8113 was set as 1. **(C)** The expression pattern of Rictor on protein level and mTORC2 activity in selected cell lines detected by western blot. **(D)** Functional interference of miR-491-3p negatively regulated Rictor protein expression and Rictor activity determined with western blot. **(E)** and **(F)** Endogenous expression pattern and functional interference of miR-491-3p negatively associated with the activity of luciferase gene linked with the 3′UTR sequence of *Rictor* and a renilla luciferase reporter for normalization. Luciferase activities were measured at 48 hours after transfection and the data was obtained from three independent experiments. The mean of the results from Tca8113 cells transfected with pMir-Wt, and cells transfected with pMir-Wt and interference control were set as 100% respectively. *p < 0.01. **p < 0.001.

### mTORC2 activity induced by Rictor enhances chemo-resistance in tongue cancer cells

Rictor is an essential component of the mTORC2 complex and it is required for mTORC2 full function. Because of the significant reduction of miR-491-3p leading to Rictor upregulation in Tca8113/PYM cells, the expression levels of Rictor and mTORC2 activity were much higher in Tca8113/PYM cells than that in Tca8113, SCC-25 and CAL-27 cell lines, which was reflected by the levels of phosphorylated Akt(Ser473), SGK1(Ser422), FOXO1(Thr24) (Figure 3C). Functional interference of miR-491-3p negatively regulated Rictor protein expressionand the mTORC2 activity (Figure 3D). Additional experiments were performed to study whether mTORC2 was involved in the development of chemo-resistance in tongue cancer cells. Tca8113/PYM cells were transfected with Rictor specific siRNAs to knockdown Rictor expression, and si-2# markedly reduced Rictor protein levels (Figure 4A). This was accompanied with decreased mTORC2 activity (Figure 4B). Importantly, downregulation of Rictor significantly sensitized Tca8113/PYM cells to PYM- and cDDP-induced growth inhibition and apoptosis (Figure 4D). Similarly, the mTOR inhibitor KU-0063794 also attenuated mTORC2 activity (Figure 4B) and sensitized Tca8113/PYM cells to the treatment of PYM and cDDP (Figure 4E). In contrast, ectopic expression of Rictor markedly increased mTORC2 activity (Figure 4B) and reduced the sensitivity of Tca8113 (Figure 4F), SCC-25 (Figure 4G) and CAL-27 (Figure 4H) cell lines to PYM and cDDP. Collectively, these data indicate that increased mTORC2 activity confers chemo-resistance in tongue cancer cells.

The article "The miR-491-3p/mTORC2/FOXO1 regulatory loop modulates chemo-sensitivity in human tongue cancer" was published in 2015. Journal: Oncotarget.

**Figure 4:** mTORC2 activation enhances chemo-resistance in tongue cancer cells **(A)** western blot result showed transfection of Rictor specific siRNAs (si-2#) efficiently downregulated Rictor protein levels, and si-2# was selected for the followed experiments. **(B)** Rictor knockdown or mTOR inhibitor KU-0063794 treatment attenuated mTORC2 activity detected by western blot. **(C)** Ectopically overexpressed Rictor with transfection of pcDNA3.1-Rictor plasmid increased mTORC2 activation measured with western blot. **(D–H)** The sensitivity of Tca8113, SCC-25 and CAL-27 cell lines to PYM and cDDP, detected by MTS assay and hochest stain respectively.

### mTORC2 signal inhibits miR-491-3p expression via FOXO1 inactivation

The mTOR signaling pathway regulates many cellular processes and is implicated in a number of pathological conditions. Thus, we next investigated the potential feedback regulation of miR-491-3p expression by mTORC2. We found that both Rcitor knockdown and treatment with an mTOR inhibitor led to significant increase of miR-491-3p expression in Tca8113/PYM cells (Figure 5A), whereas elevated expression of Rictor downregulated miR-491-3p expression in Tca8113, SCC-25 and CAL-27 cell lines (Figure 5B). It has been shown that the transcription factor FOXO1 acts as a tumor suppresser, and can be phosphorylated by Akt and SGK1 protein kinases. The phosphorylated FOXO1 (p-FOXO1) translocates from the nucleus to cytoplasm leading to transcriptional inactivation. We then analyzed the response elements of a cohort of transcription factors located within 2kb region upstream of *miR-491-3p* precursor start site using the online software “The JASPAR database”. We identified four putative FOXO1 binding sites (A, B, C, and D) within it (Figure 5C). To validate the direct association of FOXO1 with the promoter of *miR-491-3p*, we performed ChIP-qPCR assays and discovered that FOXO1 most significantly bound to site A and site D. The bindings in Tca8113/PYM cells were much lower than those in the chemo-sensitive tongue cancer cell lines (Figure 5D). Moreover, both Rictor knockdown and inhibition of mTOR activity with KU-0063794 promoted FOXO1 binding to miR-491-3p promoter at site A and site D (Figure 5E). This was accompanied with acceleration of FOXO1 transcriptional activation evidenced by the reduced p-FOXO1 (Figure 4B). In contrast, overexpression of Rictor attenuated the binding of FOXO1 to miR-491-3p promoter in Tca8113, SCC-25 and CAL-27 cell lines (Figure 4F), associated with an increased p-FOXO1 (Figure 4C). To assess whether the 2kb region indeed has promoter activity, the 2kb DNA was cloned into the pGL4 reporter plasmid. We found that the luciferase activity driven by the potential promoter of *miR-491-3p* was much higher in Tca8113, SCC-25 and CAL-27 cell lines than that in Tca8113/PYM cells (Figure 5G). In addition, both Rictor knockdown and inhibition of mTOR activity enhanced the luciferase activity (Figure 5H). Conversely, ectopic expression of Rictor not only decreased the binding of FOXO1 to the promoter of miR-491-3p (Figure 5F), it also significantly suppressed the promoter activity in Tca8113, SCC-25 and CAL-27 cell lines (Figure 5I). Taken together, these results strongly support that FOXO1 physically binds to the promoter region of *miR-491-3p* to drive its transcription. The mTORC2 signaling pathway downregulates miR-491-3p expression via inhibiting the transcriptional activation of FOXO1.

The article "The miR-491-3p/mTORC2/FOXO1 regulatory loop modulates chemo-sensitivity in human tongue cancer" was published in 2015. Journal: Oncotarget.

**Figure 5:** mTORC2 inhibits miR-491-3p expression via modulation of FOXO1 activation **(A** and **B)** Relative mean expression of miR-491-3p was determined by qRT-PCR. **(C)** A schematic representation of FOXO1 binding sites in the 2kb putative *miR-491-3p* promoter upstream of the first base of the miR-491-3p precursor start site and the first base of the 2kb set as 1. **(D–F)** ChIP-qPCR for the FOXO1 binding to the *miR-491-3p* promoter in **(D)** selected tongue cancer cell lines and (E and F) mTORC2 activity modulated cell lines by transfection of siRNA and plasmid, and mTOR inhibitor treatment respectively. **(G–I)** Luciferase reporter assay for the luciferase activity driven by miR-491-3p promoter in **(G)** selected tongue cancer cell lines and **(E)** and **(F)** mTORC2 activity modulated cell lines. *vs related control, *p* < 0.001. **vs other selected cell lines, *p* < 0.001.

### MiR-491-3p/mTORC2 axis associates with prognosis of tongue cancer patients

Given the feedback regulatory loop between miR-491-3p and mTORC2 activity identified in our cell culture studies, we wondered whether the miR-491-3p/mTORC2 axis might associate with the prognosis of tongue cancer patients. The expression levels of miR-491-3p and several components of mTORC2 signaling pathway were evaluated in clinical samples of tongue cancer patients. We performed in situ hybridizations (ISH) to detect miR-491-3p and immunohistochemical staining to examine Rictor, p-Akt(Ser473), p-SGK1(Ser422) and p-FOXO1(Thr24) in the tissues from 84 tongue cancer patients who received chemotherapy based on PYM and/or cDDP. Remarkably, ISH results demonstrated that 62 (73.81%) tongue cancer tissues exhibited relative low expression of miR-491- 3p. Among the 62 tissues, 56 of them (90.32%) showed relative high expression levels of Rictor, p-Akt(Ser473), p-SGK1(Ser422), and p-FOXO1(Thr24) (Figure 6A and 6B). On the other hand, Rictor protein was highly expressed in only 5 (22.7%) of 22 tongue cancer tissues with relative high expression of miR-491-3p (Figure 6B), suggesting an inverse correlation between miR-491-3p and Rictor in tongue cancers. Importantly, tongue cancer patients with low expression of miR-491-3p have a poorer prognosis for overall survival as compared to the patients with high expression of miR-491-3p (Figure 6C). Interestingly, high protein levels of Rictor was also predictive for a worse overall survival in tongue cancer patients (Figure 6D). Moreover, tongue cancer patients with low levels of miR-491-3p and highly expressed Rictor exhibited a significantly worse overall survival than the patients with high levels of miR-491-3p and reduced expression of Rictor (Figure 6E). These data demonstrated a negative expression pattern between miR-491–39 and Rictor or mTORC2 activity, indicating that miR-491-3p might target *Rictor* mRNA *in* vivo as well. Our clinical studies support that the miR-491-3p/mTORC2 axis associates with the prognosis of tongue cancer patients.

The article "The miR-491-3p/mTORC2/FOXO1 regulatory loop modulates chemo-sensitivity in human tongue cancer" was published in 2015. Journal: Oncotarget.

**Figure 6:** miR-491-3p expression correlated with Rictor expression and mTORC2 activity in tongue cancer, associating with prognosis of tongue cancers patients **(A)** Representative images of miR-491-3p expression detected by ISH (red staining as nucleus and blue staining as miR-491-3p level) and Rictor, p-Akt, p-SGK1 and p-FOXO1 protein levels detected by immunohistochemical staining in tongue cancer tissues (20×). **(B)** miR-491-3p expression was negatively correlated with Rictor expression in tongue cancer tissues. **(C–E)** Kaplan-Meier analysis estimated overall survival according to the miR-491-3p expression, Rictor protein level, and both miR-491-3p expression and Rictor protein level. **(F)** Schematic model depicting the miR-491-3p/Rictor-mTORC2/FOXO1 feedback regulatory loop in drug resistance of tongue cancer.

## DISCUSSION

Although significant advances have been made in the treatment of various types of cancer, drug resistance remains a major clinical obstacle. Better understanding of the underlying mechanisms is urgently needed to improve the current regimens of chemotherapy. Recent studies indicate that aberrant miRNAs expression is strongly implicated in drug resistance [6]. In the present study, miR-491-3p was found to be downregulated in PYM-induced multidrug resistant tongue cancer cells termed as Tca8113/PYM. Restored expression of miR-491-3p sensitized Tca8113/PYM cells to chemotherapy, whereas functional inhibition of miR-491-3p led to enhanced resistance of tongue cancer cells to chemotherapy. More importantly, we uncover a reduced expression of miR-491-3p in the majority of tongue cancer tissues and its downregulation significantly predicts for a poor prognosis of overall survival in tongue cancer patients. These results suggest that miR-491-3p plays a tumor suppressive role in tongue cancer. MiR-491-3p was thought to play a potential role in regulating meiotic recombination- and synapsis-related genes [18]. As to cancer, miR-491-3p was found to be downregulated in retinoblastoma cells under hypoxic condition, which is an essential feature of retinoblastoma and contributes to poor prognosis and resistance to conventional therapy [19]. Recently, Li et al. observed that miR-491-3p was downregulated in glioblastoma multiforme samples as compared to the normal brain tissues. Overexpression of miR-491-3p inhibited glioma cell invasion and proliferation and impaired the propagation of glioma stem cells [20].

The article "The miR-491-3p/mTORC2/FOXO1 regulatory loop modulates chemo-sensitivity in human tongue cancer" was published in 2015. Journal: Oncotarget.

Our current studies revealed an inverse correlation between miR-491-3p and Rictor in tongue cancer cell lines and clinical samples. The results from luciferase reporter assays confirmed that Rictor was a direct target of miR-491-3p in tongue cancer. Rictor expression status negatively associated with chemo-sensitivity in tongue cancer cell lines and with the overall survival of tongue cancer patients. Rictor is an essential component of the mTORC2 complex, and is required for its full function. The evolutionarily conserved Ser/Thr kinase mTOR (mammalian target of rapamycin) plays a pivotal role in regulating cell growth, proliferation and survival. Aberrant activation of mTOR signaling is frequently observed in many types of cancers, implicating its cancer promoting role. mTOR interacts with several proteins to form distinct complexes named mTORC1 and mTORC2. In general, mTORC1 controls cell growth by regulating mRNA translation via phosphorylation of S6K (ribosomal S6 kinase) and 4E-BP1 (4E binding protein 1), whereas mTORC2 regulates cell proliferation, survival, apoptosis, growth and actin cytoskeleton by activating Akt, PKC-α (protein kinase C-α) and SGK1 (serum-glucocorticoid-induced protein kinase-1) [21, 22]. Many gliomas overexpress the specific mTORC2 subunit Rictor. Forced expression of Rictor promotes mTORC2 assembly and activation, and endows cancer cells with increased proliferation and invasion potential [23]. Conversely, Rictor downregulation suppresses cell proliferation and migration, and promotes apoptosis in certain cancers [24, 25]. In mice, the development of prostate cancer induced by the loss of the tumor suppressor PTEN requires mTORC2 function mediated by Rictor [28]. Recent investigations indicate that several miRNAs, such as miR-152 [29], miR-218 [30], miR-424 and miR-503 [31], were involved in the dysregulation of Rictor expression. Here, we showed that Rictor was overexpressed accompanied with increased mTORC2 activation due to miR-491-3p downregulation in drug resistant tongue cancer cells. Both Rictor knockdown and mTOR inhibitor inactivated the mTORC2 downstream signaling such as Akt, SGK and FOXO1, and re-sensitized tongue cancer cells to chemotherapy. We also found the level of p-FOXO1 increased in tongue cancer cell lines and clinical samples with high Rictor and mTORC2 activity and low expression levels of miR-491-3p. FOXO1 acts as tumor suppressor and its inactivation has been documented in many types of human cancer [32]. FOXO1 activation inhibits tumor cell survival by inducing apoptosis in glioma cells through upregulating pro-apoptotic factors [33]. Our studies determined a negative feedback loop between miR-491-3p expression and mTORC2 activity through the transcription factor FOXO1. Bioinformatics analysis combined with ChIP-qPCR uncovered the physical binding of FOXO1 to the miR-491-3p promoter in tongue cancer cells. Luciferase reporter assays confirmed the direct transcriptional regulation of miR-491-3p by FOXO1.

The article "The miR-491-3p/mTORC2/FOXO1 regulatory loop modulates chemo-sensitivity in human tongue cancer" was published in 2015. Journal: Oncotarget.

In summary, as shown in Figure 6F, our studies demonstrated an important role of the negative feedback between miR-491-3p and mTORC2 signaling mediated by Rictor and FOXO1 in drug resistance of tongue cancer. It is suggested that new strategies with targeted intervention on this miR-491-3p/mTORC2 axis may significantly enhance the efficacy of chemotherapy against human tongue cancer.

## MATERIALS AND METHODS

### Cell culture and tissue specimens

The moderately differentiated human tongue squamous cell carcinoma derived cell line Tca8113 was obtained from the China Center for Type Culture Collection (Wuhan, China) and the stable PYM-resistant cell line Tca8113/PYM was previously established in our lab. The squamous cell carcinoma cell lines SCC-25 and CAL-27 were from American Type Culture Collection. Above cell lines were cultured in RPMI-1640 (Gibco, Carlsbad, CA, USA) containing 10% fetal bovine serum (Gibco) at 37°C in a humidified atmosphere containing 5% CO_2_. To maintain the resistance phenotype, 0.5mg/L PYM was added to the culture media of Tca8113/PYM cells. PYM was from PYM Harbin Bolai Pharmaceutical (Harbin, China). cDDP was from Sigma-Aldrich (Steinheim, Germany). KU-0063794 was from Selleck Chemicals (Houston, Texas, USA). Eighty-four tongue cancer tissue specimens were obtained from patients at the Affiliated Tumor Hospital of Guangzhou Medical University between March 2000–December 2006. Overall survival was computed from the day of surgery to the day of death or of last follow-up. The study was approved by the ethics committee of the Affiliated Tumor Hospital of Guangzhou Medical University.

The article "The miR-491-3p/mTORC2/FOXO1 regulatory loop modulates chemo-sensitivity in human tongue cancer" was published in 2015. Journal: Oncotarget.

### miRNA array analysis

After two weeks of culture without PYM, total RNA was isolated using Trizol reagent (Invitrogen, Carlsbad, CA, USA), and it was further purified using the RNeasy mini kit (QIAGEN, Hilden, Germany). The miRNA profiles were compared using miRCURY LNA (locked nucleic acid) microarray (Exiqon, Vedbaek, Denmark) according to the manual.

### Real-time PCR for mature miRNAs and mRNAs

miRNAs from cultured cells were isolated and purified with the miRNA isolation system (Exiqon). cDNA was generated with the miScript II RT Kit (QIAGEN), and quantitative real-time PCR (qRT-PCR) was performed by using the miScript SYBR Green PCR Kit (QIAGEN) following the manufacturer's instructions. The miRNA sequence-specific RT-PCR primers and the endogenous control RNU6 were purchased from QIAGEN. The relative quantitative expression was calculated by normalizing the results with RNU6. The total RNA was extracted according to the Trizol protocol, and cDNAs from the mRNAs were synthesized with the first-strand synthesis system (Thermo Scientific, Glen Brunie, MA, USA). Real-time PCR was carried out according to standard protocols using an ABI 7500 with SYBR Green detection (Applied Biosystems, Foster City, CA, USA). GAPDH was used as an internal control and the qRT-PCR was repeated three times. The primers for GAPDH were: forward primer 5′-ATTCCATGGCACCGTCAAGGCTGA-3′, reverse primer 5′-TTCTCCATGGTGGTGAAGACGCCA-3′; primers for Rictor were: forward primer 5′-AAGAA GCATGTCGGGGGAAT-3′, reverse primer 5′-CATGG ACCGCACTGAGGAAG-3′.

### Transfection

miR-491-3p mimics, miR-491-3p inhibitor, and relative controls were purchased from Exiqon (Vedbaek, Denmark). Cells were trypsinised, counted and seeded onto 6-well plates the day before transfection to ensure 70% cell confluence on the day of transfection. The transfection was carried out using Lipofectamine 2000 (Invitrogen, Carlsbad, CA, USA) in accordance with the manufacturer's procedure. The mimics, inhibitor and controls were used at a final concentration of 100 nM. At 36 h post-transfection, follow-up experiments were performed. The siRNAs target to Rictor and control were purchased from Santa Cruz Biotechnology (Dallas, Texas, USA). The transfection of 50 nM siRNA or control, and 4 μg of the pcDNA3.1-control and pcDNA3.1-Rictor plasmids were performed as above, 48 h later, Rictor was determined by western blot, and the experiment was repeated four times.

The article "The miR-491-3p/mTORC2/FOXO1 regulatory loop modulates chemo-sensitivity in human tongue cancer" was published in 2015. Journal: Oncotarget.

### MTS assay

The CellTiter 96 AQueous One Solution Cell Proliferation Assay kit (Promega, Madison, WI, USA) was used to determine the sensitivity of cells to PYM or cDDP. Briefly, cells were seeded in 96-well plates at a density of 4 × 10^3^ cells/well (0.2 ml/well) for 24 h before use. The culture medium was replaced with fresh medium containing PYM or cDDP at different concentrations and cells were then incubated for a further 72 h. Then, MTS (0.02 ml/well) was added. After a further 2 h incubation, the absorbance at 490 nm was recorded for each well on the BioTek Synergy 2. The absorbance represented the cell number and was used for the plotting of dose–cell number curves.

### Hoechst staining

Following transfection cells were reseeded in fresh medium in 24-well plates. After a 24 h incubation, cells were treated with or without PYM (80 mg/L) or cDDP (5 mg/L) for an additional 48 h. The cells were then stained with hoechst33528, and apoptotic cells possessing significantly smaller, condensed and fragmented nuclei, were observed using a fluorescence microscope. The apoptotic cell number was determined for at least three fields-of-view for each treatment and the apoptotic rate then calculated.

### Western blotting

Total protein was extracted from cells using RIPA buffer (Thermo Scientific, Rockford, IL, USA) in the presence of protease inhibitors (Protease Inhibitor Cocktail, Thermo Scientific). The protein concentration of lysates was measured using a BCA Protein Assay Kit (Thermo Scientific). Equivalent amounts of protein were mixed with 5 × Lane Marker Reducing Sample Buffer (Thermo Scientific), and resolved by electrophoresis in a 10% SDS–polyacrylamide gel and then transferred onto Immobilon-P Transfer Membrane (Merck Millipore, Schwalbach, Germany). The membranes were blocked with 5% non-fat milk in Tris-buffered saline and then incubated with primary antibodies followed by secondary antibody. The signal was detected on the Odyssey instrument (LI-COR Bioscience, Lincoln, Nebraska USA). Rictor, p-Akt(Ser473) and β-Actin were from Cell Signaling Technology (Danvers, MA, USA), p-SGK1(Ser422) was from Thermo Scientific. p-FOXO1(Thr24) was from Merck Millipore. The fluorescently labeled secondary antibodies were from LI-COR Bioscience.

The article "The miR-491-3p/mTORC2/FOXO1 regulatory loop modulates chemo-sensitivity in human tongue cancer" was published in 2015. Journal: Oncotarget.

### Luciferase reporter assay

For miRNA luciferase reporter assay: The DNA sequences with each 50 base at up-and downstream of miR-491-3p binding site in the 3′UTR of Rictor (as wildtype version) and DNA sequences with 7 bases deleted in the miR-491-3p binding site (as mutant version), were synthesized with restriction sites for SpeI and HindIII located at both ends of the oligonucleotides for further cloning, and subsequently cloned into pMir-Report plasmid downstream of firefly luciferase reporter gene. Cells were seeded in 96 well-plates and co-transfected with pMir-Report luciferase vector, pRL-TK Renilla luciferase vector and miR-491-3p mimics or inhibitor using Lipofectamine 2000 (Invitrogen). For promoter activity assay: To determine whether FOXO1 regulates the promoter activity of miR-491-3p, a two kilobase region upstream of the miR-491-3p precursor starting site was cloned into the pGL4-reporter vector upstream of the luciferase gene. Cells were seeded in 96-well plates and co-transfected with the pGL4-reporter vector and the pRL-TK Renilla luciferase vector with or without the pcDNA3.1-Rictor vector using. After transfection of 48 h, luciferase activity was determined using a Dual-Luciferase Reporter Assay System (Promega) on the BioTek Synergy 2. The Renilla luciferase activity was used as internal control and the firefly luciferase activity was calculated as the mean ± SD after being normalized by Renilla luciferase activity.

### ChIP-qPCR

The ChIP assay was performed using the EZ-CHIP^TM^ chromatin immunoprecipitation kit (Merck Millipore). Briefly: Chromatin proteins were cross-linked to DNA by addition of formaldehyde to the culture medium to a final concentration of 1%. After a 10 min incubation at room temperature, the cells were washed and scraped off in ice-cold phosphate-buffered saline (PBS) containing Protease Inhibitor Cocktail II. Cells were pelleted and then resuspended in lysis buffer containing Protease Inhibitor Cocktail II. The resulting lysate was subjected to sonication to reduce the size of DNA to approximately 200–1000 base pairs in length. The sample was centrifuged to remove cell debris and diluted ten-fold in ChIP dilution buffer containing Protease Inhibitor Cocktail II. Then 5 μg of anti-RNA Polymerase antibody (positive control, included with the kit), or anti-FOXO1 antibody (cell signal technology) were added to the chromatin solution and incubated overnight at 4°C with rotation. After antibody incubation, protein G agarose was added and the sample incubated at 4°C with rotation for an additional 2 h. The protein/DNA complexes were washed with Wash Buffers four times and eluted with ChIP Elution Buffer. Cross-links were then reversed to free DNA by the addition of 5 M NaCl and incubation at 65°C for 4 h. The DNA was purified according to the manufacturer's instructions. 50 μl of DNA was obtained for each treatment. 2 μl of DNA from each group was used as a template for PCR. Primers for the miR-491-3p promoter containing putative FOXO1 binding sites were as follows, sense: 5′-GAGATCAAGGGAACTTGGTTTTTC-3′, antisense: 5′-CAGGGCCCTCTAGGTCACC-3′ (for site A); sense: 5′-GTTAATCTAGGGCTGTTTATTGACAT-3′, antisense: 5′-ATCCCATTTCCATGAAGCACTGAAC-3′ (for site B); sense: 5′-GGTTTGAATTTCCAAATTCTCT TATCC-3′, antisense: 5′-GTTCAGTTAAAAATCC ACAGAACAGG-3′ (for site C); sense: 5′-GACATGG AAAGCAAATATT TGAAATTG-3′, antisense: 5′-GAGGGGCCTACTAGTT AATCAAG-3′ (for site D). Primers for the human GAPDH gene: sense, 5′-TACTAGCGGTTTTACGGGCG-3′, antisense, 5′-TCGAACAGGAGGAGCAGAGAGCGA-3′. The PCR conditions were as follows: 1 cycle of 95°C for 5 min; 40 cycles of 95°C for 20 s, 60°C for 30 s, and 72°C 30 s; and 1 cycle of 72°C for 10 min. The results were calculated by normalizing to the positive control, and relative quantization values were calculated using % positive control = 2^(−ΔCt [(Ct [FOXO1] − (Ct [positive control]]) method.

The article "The miR-491-3p/mTORC2/FOXO1 regulatory loop modulates chemo-sensitivity in human tongue cancer" was published in 2015. Journal: Oncotarget.

### miRNA In Site Hybridizations (ISH) assay

The miR-491-3p expression in tongue cancer samples was detected by In Site Hybridizations (ISH) with kit from Exiqon (Vedbaek Denmark) according to the manufacturer's instructions. Briefly, the sections were dried at 65°C for 3 h and then deparaffinized in xylene and ethanol at room temperature (RT) followed with a 10 min incubation with proteinase-k at 37°C. After dehydration in ethanol, sections were hybridizated with 40 nM double-DIG LNA™ miR-491-3p probe 55°C for 1 h. After wash in SSC buffer at hybridization temperature and incubation with blocking solution for 15 min, the anti-DIG reagent sheep anti-DIG-AP (Roche, Mannheim, Germany) was applied and incubated for 60 min at RT. After wash in PBST, the sections were incubated with AP substrate NBT-BCIP (Roche) for 2 h at 30°C and incubated in KTBT buffer to stop reaction. Then the nuclear counter stain Nuclear Fast Red™ (Vector labs, Burlingame, CA) was applied for 1 min for nuclear counter staining, and slides were rinsed in tap water for 10 min. after dehydrated in ethanol and mounted, the sections were investigated and analyzed under microcopy.

### Immunohistochemistry

A tissue array containing 84 human tongue cancer specimens was cut into 4-μm sections. The sections were dried at 62°C for 2 h and then deparaffinized in xylene and rehydrated using a series of graded alcohol washes. The tissue slides were then treated with 3% hydrogen peroxide in methanol for 15 min to quench endogenous peroxidase activity and antigen retrieval then performed by incubation in 0.01 M sodium cirate buffer (pH 6.0) and heating using a microwave oven. After a 1 h preincubation in 10% goat serum, the specimens were incubated with primary antibody overnight at 4°C. The tissue slides were treated with a non-biotin horseradish peroxidase detection system according to the manufacturer's instruction (DAKO, Glostrup, Denmark). Two different pathologists evaluated the immunohistological samples.

The article "The miR-491-3p/mTORC2/FOXO1 regulatory loop modulates chemo-sensitivity in human tongue cancer" was published in 2015. Journal: Oncotarget.

### Statistical analysis

All statistical analyses were performed with SPSS statistical software (version 21.0; IBM). Survival curves were constructed using the Kaplan–Meier method and analyzed by the log-rank test. Significant prognostic factors identified by univariate analysis were entered into multivariate analysis using the Cox proportional hazards model. The Student's *t*-test was used for comparisons and the Pearson correlation test (two-tailed) was used to investigate the correlation between miR-491-3p and Rictor protein level. Statistical significance was defined as *p* < 0.05.
